The article "Different Vancomycin Immunoassays Contribute to the Variability in Vancomycin Trough Measurements in Neonates" was published in 2016. Journal: Biomed Res Int.

# Different Vancomycin Immunoassays Contribute to the Variability in Vancomycin Trough Measurements in Neonates

**DOI:** 10.1155/2016/1974972

**Published:** 2016-08-21

**Authors:** Janko Samardzic, Anne Smits, Isabel Spriet, Ivan Soldatovic, Andrew Atkinson, Milica Bajcetic, John N. Van Den Anker, Karel Allegaert

**Affiliations:** ^1^Institute of Pharmacology, Clinical Pharmacology and Toxicology, Medical Faculty, University of Belgrade, 11000 Belgrade, Serbia; ^2^Division of Pediatric Pharmacology and Pharmacometrics, University of Basel Children's Hospital, 4056 Basel, Switzerland; ^3^Department of Development and Regeneration, KU Leuven, 3000 Leuven, Belgium; ^4^Neonatal Intensive Care Unit, University Hospitals Leuven, 3000 Leuven, Belgium; ^5^Clinical Pharmacology and Pharmacotherapy, Department of Pharmaceutical and Pharmacological Sciences, KU Leuven and Pharmacy Department, University Hospitals Leuven, 3000 Leuven, Belgium; ^6^Medical Faculty, University of Belgrade, 11000 Belgrade, Serbia; ^7^Clinical Pharmacology Unit, University Children's Hospital, 11000 Belgrade, Serbia; ^8^Division of Pediatric Clinical Pharmacology, Children's National Medical Center, Washington, DC 20010, USA; ^9^Intensive Care and Department of Pediatric Surgery, Erasmus MC Sophia Children's Hospital, 3000 CB Rotterdam, Netherlands

## Abstract

Substantial interassay variability (up to 20%) has been described for vancomycin immunoassays in adults, but the impact of neonatal matrix is difficult to quantify because of blood volume constraints in neonates. However, we provide circumstantial evidence for a similar extent of variability. Using the same vancomycin dosing regimens and confirming similarity in clinical characteristics, vancomycin trough concentrations measured by PETINIA (2011-2012, *n* = 400) were 20% lower and the mean difference was 1.93 mg/L compared to COBAS (2012–2014, *n* = 352) measurements. The impact of vancomycin immunoassays in neonatal matrix was hereby suggested, supporting a switch to more advanced techniques (LC-MS/MS).

## 1. Introduction

Vancomycin, a glycopeptide antibiotic, is commonly used in neonatal intensive care units (NICUs) for the treatment of late onset sepsis and catheter-related infections [1]. In adults, a ratio of the 24-hour area under the curve (AUC_0–24_) divided by the minimum inhibitory concentration (MIC) for a given pathogen ≥ 400 is considered to be the optimal predictor of vancomycin efficacy for invasive methicillin-resistant staphylococci (MRSA) respiratory infections. Vancomycin serum concentrations are widely used as a surrogate marker for AUC, aiming to achieve target trough concentrations between 10 and 15 mg/L during intermittent intravenous administration [2].

The article "Different Vancomycin Immunoassays Contribute to the Variability in Vancomycin Trough Measurements in Neonates" was published in 2016. Journal: Biomed Res Int.

Large interindividual variability in vancomycin pharmacokinetics (PK) within the neonatal population is well-known and is only in part explained by covariates such as weight, age, or serum creatinine [3, 4]. Since therapeutic drug monitoring (TDM) is clinically useful for drugs that have a known relationship between measured bodily fluid concentration and therapeutic effect, neonates with their rapid developmental changes in pharmacokinetic parameters will benefit from vancomycin TDM [5]. However, even if TDM is implemented, the immunoassays currently used to quantify vancomycin concentrations may differ because of differences in matrix. Cross-validation of different published PK models on vancomycin in neonates from different NICUs failed [6]. Clinicians do not take into account that routine vancomycin quantification by commercial immunoassays can indeed show substantial differences, and this is an important clinical argument in support of a switch towards LC-MS/MS methodologies [7–10].

While this phenomenon is obviously not limited to neonatal matrix, the relevance may be population specific because of differences in plasma composition (e.g., concentration of albumin, immunoglobulins like IgA, and bilirubin) [7, 8]. Current recommendations do not take into account that routine plasma vancomycin quantification by commercial immunoassays can show substantial between-method differences. Next to standardization issues, immunoassays can also lack specificity. Cross-reacting substances such as vancomycin degradation products have been described to interfere with some immunoassays [7–10].

Unfortunately, there are no data on the interassay differences in neonatal matrix, likely due to blood volume constraints. Since the blood samples are of very limited quantity in neonates, it is not feasible to analyze different between-assay differences in a paired study design as applied in adult samples [7–9]. In an attempt to provide circumstantial evidence, we explored the impact of between-assay differences on the variability in vancomycin serum trough levels measured in neonates treated in a single neonatal intensive care unit (NICU) following a switch in immunoassay (PETINIA to COBAS).

## 2. Design and Methods

### 2.1. Study Population, Clinical Data Collection, and Ethics

Vancomycin trough concentrations measured in neonates and young infants treated with intravenous vancomycin, mainly for (suspected) late onset sepsis (>72 hours after birth), in the NICU of the University Hospitals Leuven, Belgium, between June 2011 and December 2014, were considered for inclusion in this retrospective study. Our patient population consisted of preterm and term neonates, who needed specialized care related to infections and prematurity. Clinical characteristics at birth (birth weight [BW] in grams; gestational age [GA] in weeks) and characteristics at the moment of TDM (postmenstrual age [PMA] in weeks, postnatal age [PNA] in days, weight at inclusion [WT] in grams, serum creatinine (mg/dL), serum albumin (g/L), and serum trough vancomycin concentration (mg/L)) were extracted from the patient files. Results were excluded if data regarding vancomycin prescription could not be obtained or in case of an administration or sampling time error. The ethics board of our hospital approved the study protocol.

The article "Different Vancomycin Immunoassays Contribute to the Variability in Vancomycin Trough Measurements in Neonates" was published in 2016. Journal: Biomed Res Int.

### 2.2. Vancomycin Indication, Administration, TDM Collection, and TDM Assays

Vancomycin (Vancocin®, Elly Lilly, Brussels, Belgium) combined with amikacin is used as standard therapy for (suspected) late onset sepsis. Administration occurs as an intravenous infusion over 60 minutes. The vancomycin dosing regimen was based on PMA and serum creatinine, irrespective of the vancomycin assay used [4]. As part of routine clinical care trough samples for TDM were collected at the end of the dosing interval, in most cases 24–72 hours after treatment was initiated. Subsequent trough TDM samples during the same course were collected based on the decision of the attending physician. All samples during the first vancomycin treatment course are included.

During the study period, two different vancomycin immunoassays were applied consecutively. The vancomycin serum trough concentrations were measured either by a particle-enhanced turbidimetric inhibition immunoassay method (Siemens Dimension; Dade Behring, Deerfield, Illinois, PETINIA) or by an enzyme multiplied immunoassay technique (Cobas c702; Roche Diagnostics, Germany, COBAS). In November 2012, the assay was changed from PETINIA to COBAS throughout the entire hospital for logistic, nonclinical reasons. The hospital laboratory has a quality system that conforms to ISO15189. This implies that clinical interchangeability of results is verified when changing from one assay to another. To avoid censoring of concentrations below the lower limit of quantification (2 mg/L), these concentrations were replaced by a lower limit of quantification/2 (1 mg/L) [11]. Throughout this study interval, an enzymatic technique (Cobas c702 module) was used to quantify serum creatinine concentrations, so issues on Jaffe versus enzymatic creatinine assays do not apply [12].

### 2.3. Data Analysis and Statistics

The data were analyzed by Student's *t*-test and Mann-Whitney *U* test, as appropriate. General linear modelling was performed to assess significant differences between both groups, when adjusting for confounding factors. Since vancomycin serum concentrations had a small deviation of distribution, these were transformed using logarithmic transformation to obtain a normal distribution. Data were analyzed in SPSS 20.0 (IBM corp.) and a *p* value < 0.05 was considered statistically significant.

The article "Different Vancomycin Immunoassays Contribute to the Variability in Vancomycin Trough Measurements in Neonates" was published in 2016. Journal: Biomed Res Int.

## 3. Results and Discussion

Our dataset comprised 313 patients with 752 vancomycin trough TDM observations: 400 observations were assayed with PETINIA and 352 with COBAS. Both cohorts had comparable clinical characteristics and only differences for serum albumin concentration were documented (Table 1).

We observed a significant difference between the vancomycin trough concentrations using two different immunoassays: PETINIA versus COBAS (*F* = 7.695; *p* = 0.006, Figure 1). When adjusting for serum albumin concentration and creatinine levels as critical covariates, the difference in vancomycin concentration between cohorts remained statistically significant (*F* = 4.567, *p* = 0.033; *F* = 4.302; *p* = 0.038, resp.). According to these results, it was shown that the vancomycin assay used was a significant predictor of vancomycin serum concentration. Overall, immunoassays PETINIA and COBAS yielded significantly different vancomycin trough concentrations when adjusting for covariates and the mean difference was 1.93 mg/L. The vancomycin serum trough concentrations measured by PETINIA were 20% lower than those measured by COBAS (Figure 1).

Vancomycin dosing strategies in neonates are mostly based on postmenstrual and postnatal age, and they also take into account the developmental changes in volume of distribution and renal function as the most important covariates influencing vancomycin clearance [2]. However, the clinical significance of different analytical methods for serum vancomycin concentration was only recently suggested in neonates [6]. Between-assay studies in neonatal matrix are hampered by the blood volume needed to perform multiple between-assay studies, but we here provided circumstantial evidence of the relevance and the impact.

This provides further evidence that dosage individualization should not only consider clinical characteristics but also be tailored to the method of vancomycin quantification in neonates [6, 9]. We hereby speculate that this reflects the fact that immunoglobulin M (IgM) or IgA affects vancomycin concentration measured by PETINIA [10]. This might at least in part explain between-assay differences in the neonatal plasma matrix. Importantly, the relevance goes beyond our single institution, as illustrated by Zhao et al.: the transferability of published models of vancomycin pharmacokinetics to different clinical settings in part related to the use of conversion factors to “correct” for differences in vancomycin immune assays used [6].

The article "Different Vancomycin Immunoassays Contribute to the Variability in Vancomycin Trough Measurements in Neonates" was published in 2016. Journal: Biomed Res Int.

The impact of vancomycin immunoassays in neonatal matrix was hereby suggested, providing additional support to switch to more advanced techniques (LC-MS/MS) to avoid both the matrix related differences between immunoassays and to lower the blood volume needed to quantify vancomycin in neonatal samples. Until then, clinicians taking care for neonates should consider the impact of immunoassays on vancomycin levels and targets. Similar, researchers should consider including neonatal samples in their assay comparison and assay development. Obviously and because of the limitations (sample volume) and ethical constrains in neonates, such studies should first be done using samples for adult patients. Matrix effects (ion suppression/enhancement) should hereby be considered, since this is a well-observed phenomenon in analyses of biological matrices by high-performance liquid chromatography-mass spectrometry (LC-MS) [13]. This should be followed by subsequent hypothesis testing, validation, or confirmation in neonatal matrix. Pooling of neonatal samples is hereby one of the approaches to further reduce this burden.

## Figures and Tables

**Figure 1:** Vancomycin serum trough concentrations (mg/L) determined by two different immunoassays: PETINIA versus COBAS, presented as box plots (Mann-Whitney *U* test, *p* < 0.05).

**Table 1:** Clinical characteristics of studied patients. Data are provided by mean and standard deviation (SD).

	Mean	SD	*p* value
Gestational age (weeks)			
PETINIA	31.91	5.17	0.635
COBAS	31.71	5.27	

Birth weight (g)			
PETINIA	1,779.48	991.96	0.182
COBAS	1,906.91	1,143.24	

Weight at inclusion (g)			
PETINIA	2,066.77	1,101.14	0.233
COBAS	2,220.59	1,288.11	

Postmenstrual age (weeks)			
PETINIA	34.77	5.98	0.766
COBAS	34.61	6.00	

Postnatal age (days)			
PETINIA	20.98	22.31	0.951
COBAS	22.13	23.38	

Creatinine (mg/dL)			
PETINIA	0.47	0.19	0.052
COBAS	0.52	0.24	

Albumin (g/dL)			
PETINIA	31.13	5.09	<0.001
COBAS	29.42	4.71	
